# Ultrasonographic findings in a cow with abomasal lymphosarcoma: Case report

**DOI:** 10.1186/1746-6148-7-20

**Published:** 2011-05-25

**Authors:** Ueli Braun, Charlotte Schnetzler, Martina Dettwiler, Titus Sydler, Sven Meyer, Christian Gerspach

**Affiliations:** 1 Department of Farm Animals, Vetsuisse Faculty, University of Zurich, Winterthurerstrasse 260, CH-8057 Zurich, Switzerland; 2 Institute of Veterinary Pathology, Vetsuisse Faculty, University of Zurich, Winterthurerstrasse 260, CH-8057 Zurich, Switzerland; 3 Veterinary Clinic Dr. Andreas Mittelholzer, Gaiserstrasse 15, 9050 Appenzell, Switzerland

## Abstract

**Background:**

This case report describes the clinical and ultrasonographic findings in a Swiss Braunvieh cow with lymphosarcoma of the abomasum.

**Case Presentation:**

The main clinical findings were vomiting in response to eating and melena. The results of serum biochemistry and rumen fluid analysis were indicative of abomasal reflux syndrome. The main ultrasonographic findings were two enlarged lymph nodes caudal to the reticulum and a severely enlarged abomasum with thickening of the abomasal wall and folds. Based on all the findings, pyloric stenosis caused by lymphosarcoma was tentatively diagnosed and later confirmed at postmortem examination.

**Conclusions:**

This is an interesting case, which broadens the spectrum of abomasal reflux syndrome.

## Background

Diseases affecting the abomasum in cattle include left and right abomasal displacement, volvulus, ulcers and parasite infestation [1]. Neoplasia of the abomasum is rare in cattle. The adult or enzootic form of lymphosarcoma, which may be spontaneous or associated with enzootic bovine leukosis, is the most common tumour affecting this organ [1]. Less common tumours include carcinoma, sarcoma and adenoma [1]. Lymphosarcoma causes thickening of the abomasal wall, which leads to progressive impairment of passage of ingesta, ulcers, haemorrhage, melena, anaemia and occasionally abomasal reflux and hypochloraemic alkalosis [2]. Diagnosis of abomasal lymphosarcoma may be difficult when peripheral lymphadenopathy is absent; this occurred in 46% of 112 cases described [3]. Clinical signs such as anorexia, weight loss and melena are suggestive of an abomasal ulcer but cannot be used to determine the cause. Lymphoblasts in a peripheral blood smear are indicative of lymphosarcoma but are seen in only approximately 10% of cases [3]. Thus, there is clearly a need for a more efficient method of diagnosis. In a recent case presented to our hospital because of melena, round to oval structures were seen via ultrasonography caudal to but not in direct contact with the reticulum. The lesions could not be interpreted and the cow was euthanased because of lack of response to treatment for possible bleeding abomasal ulcer. Postmortem examination revealed malignant lymphosarcoma of the abomasum, and the unidentified structures seen on ultrasonography were enlarged lymph nodes. A second cow with similar ultrasonographic findings was recently referred to our clinic. The structures caudal to the reticulum were identified as enlarged lymph nodes, and a tentative diagnosis of lymphosarcoma of the abomasum was made and confirmed at necropsy. The purpose of this case report was to describe the clinical and ultrasonographic findings in this cow.

## Case presentation

A 3.3-year-old Swiss Braunvieh cow, which was three months pregnant, was referred to our clinic because of poor appetite and vomiting in response to eating. The cow had not responded to treatment with a magnet, a non-steroidal anti-inflammatory drug, neostigmine and vitamin B. The general condition and demeanour of the cow were mildly impaired, and there was reduced skin turgor, mild sunken eyes, scleral injection and excessive salivation. The heart rate was decreased at 48 bpm, the respiratory rate was 28 breaths per minute and the rectal temperature was 38.5°C. On transrectal examination, the rumen was distended. The faeces had a porridge-like consistency and were dark olive in colour and positive for occult blood (hemo FEC®, Roche Diagnostics). After physical examination, the cow was placed in a stall for observation. She hesitated before apprehending, chewing and swallowing hay. This was followed a few minutes later by salivation and retching. During the ensuing 15 minutes, the cow vomited liquid and foul-smelling ruminal contents.

The cow had leukocytosis with neutrophilia (15'300 leukocytes/μl; normal 5'000 to 10'000 leukocytes/μl). Urea (13.0 mmol/l; normal 2.4 to 6.5 mmol/) and creatinine concentrations (119 μmol/l; normal 55 to 103 μmol/l) and the activities of glutamate dehydrogenase (GLDH; 30.5 U/l; normal 4 to 18 U/l) and sorbitol dehydrogenase (SDH; 67.8 U/l; normal 4 to- 7 U/l) were increased. Serum potassium (3.7 mmol/l; normal 4.0 to 5.0 mmol/l) and chloride concentrations (93 mmol/l; normal 100 to 105 mmol/l) were decreased and the concentration of inorganic phosphorus (3.7 mmol/l; normal 1.3 to 2.4 mmol/l) was increased. The chloride concentration of ruminal juice was markedly increased at 72 mmol/l (normal 15 to 30 mmol/l). Blood gas analysis revealed compensated metabolic alkalosis with a base excess of +9.1 mmol/l (normal -2 to + 2 mmol/l) and a pH of 7.45 (normal 7.40 to 7.50). An ELISA for bovine leukemia virus (CHEKIT® BLV-ELISA kit, IDEXX Switzerland) was negative.

Endoscopic examination of the oesophagus and radiographic examination of the reticulum revealed no abnormal findings. Ultrasonographic examination of the reticulum (LOGIQ 7, GE Healthcare) using a 5.0 MHz convex transducer with a penetration depth of 10 cm showed reticular hypermotility with five normal biphasic contractions per 3 minutes (normal 3 to 4 contractions) [4]. Two large oval heterogeneous structures measuring 4.5 × 5.2 cm were seen caudal to the reticulum and were thought to be lymph nodes (Figure 1). Scanning of the right side revealed that the abomasum extended to the cranial flank because of severe dilatation. The abomasal contents were hypoechogenic and the wall and folds of the abomasum were thicker than normal. The pylorus was seen in the cranial flank region at the level of the costochondral junction (Figure 2). It was positioned horizontally and was increased in size with a diameter of 10 cm.

**Figure 1:** **Ultrasonogram of enlarged lymph nodes**. Ultrasonogram of two markedly enlarged lymph nodes caudal to the reticulum in a Swiss Braunvieh cow with lymphosarcoma of the abomasum. The image was obtained from the left paramedian region lateral to the sternum using a 5.0-MHz convex transducer. 1 Ventral abdominal wall, 2 Diaphragm, 3 Reticulum, 4 Anterior ventral blind sac of rumen, 5 Lymph nodes, Cr Cranial, Cd Caudal.

**Figure 2:** **Ultrasonogram of the enlarged pylorus**. Ultrasonogram of the enlarged pylorus in a Swiss Braunvieh cow with lymphosarcoma of the abomasum. The pylorus contains ingesta and the thickness of its wall is increased. The image was obtained from the cranial right flank at the level of the costochondral junction using a 5.0-MHz convex transducer. 1 Lateral abdominal wall, 2 Thickened wall of pylorus, 3 Ingesta in pylorus, Ds Dorsal, Vt Ventral.

The clinical findings were suggestive of pyloric stenosis causing vomiting. Based on previous experience involving a cow with similar ultrasonographic findings (enlarged lymph nodes caudal to reticulum, thickened abomasal wall and folds) a tentative diagnosis of lymphosarcoma of the abomasum was made. The cow was euthanased because of a grave prognosis, and necropsied. The rumen was severely distended with liquid contents. The abomasum was 107 cm long and dilated, and the mucosa had multiple superficial ulcers. The wall of the abomasum and pylorus was severely thickened and very firm (Figures 3 and 4). The omasum was also dilated and its serosa had nodular lesions. Several gastrointestinal lymph nodes and those of the lungs and spleen were greatly enlarged, as were the two lymph nodes seen during ultrasonography (Figure 5). The tentative diagnosis of lymphosarcoma was confirmed via histological examination of the abomasum, omasum and various lymph nodes. There was infiltration of all layers of the abomasal wall (tunica mucosa, submucosa and muscularis), the serosa of the omasum and the enlarged lymph nodes with a homogeneous population of round lymphoblasts, which were 10 to 15 μm in diameter and had little cytoplasm and a round to oval nucleus (Figure 6). The chromatin of the nuclei was vesicular and nucleoli occurred sporadically. There were moderate numbers of mitotic figures, some of which were atypical. The tumour cells were surrounded by a sparse fibrovascular stroma. Immunohistochemical testing showed that the lymphoblasts were CD3-positive (and CD79a-negative) und thus were derived from T-lymphocytes. This clearly excludes false negativ ELISA since BLV causes B-cell lymphoma.

**Figure 3:** **Postmortem specimens of abomasal folds**. Postmortem specimens of severely thickened, ulcerated and erythematous abomasal folds in a Swiss Braunvieh cow with lymphosarcoma of the abomasum.

**Figure 4:** **Postmortem specimen of the pylorus**. Postmortem specimen of the pylorus showing a severely thickened mucous membrane in a Swiss Braunvieh cow with lymphosarcoma of the abomasum.

**Figure 5:** **Postmortem specimens of lymph nodes**. Postmortem specimens of severely enlarged lymph nodes, which were located caudal to the reticulum in a Swiss Braunvieh cow with lymphosarcoma of the abomasum.

**Figure 6:** **Histology of the abomasum**. Histological section of the abomasum of a Swiss Braunvieh cow with lymphosarcoma. There is infiltration of large round lymphoblasts measuring 10 to 15 μm with sparse cytoplasm and round to oval nuclei in the tunica submucosa and tunica muscularis. The chromatin appears vesicular and there are sporadic nucleoli. Haematoxylin and eosin stain.

Vomiting is uncommon in ruminants and represents a clinical sign that is of utmost concern to the owner and veterinarian. There are numerous causes of vomiting in cattle [1]. In its chronic form, vomiting may be associated with localised diseases of the alimentary tract, such as actinobacillosis of the tongue, stomatitis, pharyngitis, oesophagitis, mediastinal abscess, traumatic reticuloperitonitis and actinobacillosis of the reticulum [1]. Rumen overload associated with ileus of the forestomach/abomasal complex, frothy bloat and other disorders may also cause vomiting [1]. In the present case, it was relatively easy to make a symptomatic diagnosis of pyloric stenosis. The increased chloride concentration of rumen fluid together with the hypochloraemic and hypokalaemic compensated alkalosis were indicative of abomasal reflux syndrome, which resulted in ruminal dilatation and subsequent, overflow' vomiting as described [1]. A trigger such as feed intake, which was seen in the present case, is thought to initiate a ruminal contraction that leads to abrupt vomiting [1]. The enlarged abomasum was indicative of stenosis of the pylorus and melena suggested ulcers as the cause. The crucial criterion for the tentative diagnosis of lymphosarcoma was the enlarged lymph nodes seen caudal to the reticulum via ultrasonography. This same finding was seen in a previous case of lymphosarcoma confirmed at necropsy. Although a definitive antemortem diagnosis was not possible in that case, we were confident that the changes were not associated with traumatic reticuloperitonitis. The latter is associated with fibrinous deposits and abscessation, which have a different ultrasonographic appearance [5]. In both cases, the peripheral lymph nodes were normal on palpation. In sporadic lymphosarcoma, approximately half the cases do not have peripheral lymphadenopathy [3]. Abomasal lymphosarcoma is often accompanied by ulcers [2,6] and it is important to differentiate between the two conditions because treatment may be indicated for ulcers but not for lymphosarcoma. Results indicate that ultrasonography is the only practical method for diagnosing abomasal lymphosarcoma. The ultrasonographic changes noted in the abomasum were not striking in appearance and were limited to focal/diffuse thickening of the wall and folds. In a cow with multicentric lymphoma, which also involved the abomasum, the abomasal wall was disrupted by a cauliflower-shaped mass of mixed echogenicity [7]. In four cows with abomasal lymphoma, the most prominent finding was thickening of the abomasal and pyloric wall [8]. In three of these cows, the diagnosis was confirmed using ultrasound-guided fine needle biopsy. It is likely that an antemortem diagnosis could also have been made in our patient using this diagnostic technique. The present case was sporadic lymphosarcoma [2], which is not caused by a virus and mainly affects calves and young cattle. The enzootic form caused by bovine leukemia virus only occurs in adult cattle. All the recently published cases of lymphosarcoma in Switzerland involved the sporadic form [9-11] as did various cases of thymic lymphoma [12] and cutaneous lymphoma [13].

## Conclusions

This is an interesting case, which broadens the spectrum of abomasal reflux syndrome.

## Competing interests

The authors declare that they have no competing interests.

## Authors' contributions

UB supervised the clinical and ultrasonographic examination, reviewed the literature and prepared the manuscript. CS, SM and CG carried out the clinical and ultrasonographic examination. MD and TS performed the postmortem examination. All authors read and approved the final manuscript.
